The article "Clinical Nursing Pathway Improves Therapeutic Efficacy and Quality of Life of Elderly Patients with Acute Myocardial Infarction" was retracted in 2023. Reasons: unreliable results or conclusions; lack of ethics approval or compliance; concerns about the data; concerns about the peer review.

# Clinical Nursing Pathway Improves Therapeutic Efficacy and Quality of Life of Elderly Patients with Acute Myocardial Infarction

**DOI:** 10.1155/2022/3484385

**Published:** 2022-03-15

**Authors:** Yumei Zhang, Guichun Chen, Dandan Huang, Shue Luo

**Affiliations:** Cardiovascular Department (N21 District), The First Hospital of Quanzhou Affiliated to Fujian Medical University, Quanzhou, 362000 Fujian, China

## Abstract

**Purposes:**

To clarify the impacts of clinical nursing pathway (CNP) on therapeutic efficacy and quality of life (QOL) of senile acute myocardial infarction (AMI) patients.

**Methods:**

The clinical records of 177 elderly AMI patients who received treatment in the First Hospital of Quanzhou Affiliated to Fujian Medical University were retrospectively studied. They were assigned into the control group (the Con; *n* = 79; from June 2019 to January 2020) and the research group (the Res; *n* = 98; from February 2020 to July 2020). Emergency percutaneous coronary intervention (PCI) was performed in all the cases. Additionally, the Con and the Res were given routine care and CNP, respectively. The two groups were compared in total emergency treatment time, hospital stay, medical expenses, recurrence rate of myocardial infarction (MI), overall response rate (ORR), incidence of complications, cardiac function indexes, negative mood scores, QOL, and nursing satisfaction.

**Results:**

The ORR was higher, and the incidence of complications was lower in the Res versus the Con; the Res presented significantly less emergency treatment time and hospitalization and statistically lower medical expenses and recurrence rate of MI; the Res outperformed the Con in cardiac function indexes, alleviation of negative mood, QOL, and nursing satisfaction.

**Conclusions:**

While effectively improving clinical efficacy and reducing the incidence of complications, CNP can relieve the bad mood of elderly patients with AMI and improve their cardiac function, QOL, and nursing satisfaction, which is worthy of clinical promotion.

## 1. Introduction

As a severe cardiovascular disease, acute myocardial infarction (AMI) refers to the sharp decrease or disturbance of coronary artery blood supply triggered by coronary artery diseases, resulting in severe and persistent acute myocardial ischemia leading to myocardial necrosis [1]. In recent years, there is a rising incidence of AMI at younger ages, with a mortality up to 10%-13%, which makes AMI the leading cause of cardiac death [2]. The disease is characterized by rapid progression and fast onset, with the clinical presentations of arrhythmia, cardiogenic shock, and persistent retrosternal pain, posing a grave threat to the life safety of patients [3]. Emergency percutaneous coronary intervention (PCI) is currently the preferred treatment for AMI, which can open and dredge blood vessels as soon as possible to restore blood flow, thus limiting the range of infarcted myocardium and significantly improving the prognosis of patients [4, 5]. However, emergency patients may still experience coronary restenosis and ischemia after PCI [6]. It is shown that perioperative nursing care of patients with AMI undergoing interventional therapy directly affects the success of surgery and is the key to reducing complications and improving the success rate of rescue; hence, it carries huge clinical implications for seeking a safe and efficient care mode to improve the outcome and curative effect of AMI patients [7].

Clinical pathway, as an optimized, simplified, and synergistic management, is a standardized diagnosis, treatment, and nursing model that can effectively restrain the growth of medical expenses and effectively improve medical and nursing levels [8]. Therefore, exploring the implementation methods of clinical pathway in line with China's national conditions carries great implications for improving medical quality, reducing medical expenses, shortening length of hospitalization, promoting the rational utilization of medical resources, and enhancing the competitiveness of hospitals [9]. Clinical nursing pathway (CNP) is a comprehensive and deep-rooted new medical care model, which takes a specific disease as the research object and formulates scientific and reasonable nursing plans based on previous nursing experience to make nursing work more active and continuous [10]. With the goal of reducing the length of stay (LOS) and improving the treatment efficiency, CNP can effectively resolve patients' clinical symptoms and improve their quality of life (QOL) [11]. The innovation of this study lies in that we adopt a novel and comprehensive nursing mode for elderly patients with AMI, which is more standardized and efficient than the conventional one.

Herein, CNP was given to senile AMI patients, aiming at clarifying its impact on therapeutic efficacy and patients' QOL.

## 2. Materials and Methods

### 2.1. Baseline Data

The retrospective study enrolled 177 senile AMI cases who received treatment in the First Hospital of Quanzhou Affiliated to Fujian Medical University from June 2019 to July 2020. Among them, 79 patients recruited between June 2019 and January 2020 were assigned to the control group (the Con) and given routine nursing, while 98 enrolled from February 2020 to July 2020 were included in the research group (the Res) and given CNP. The male-to-female ratio and the mean age were 43 : 36 and 65.54 ± 3.74 years (range: 60-72) in the Con and 54 : 44 and 66.02 ± 3.82 years (range: 62-75) in the Res, respectively. This study was ethically ratified by the First Hospital of Quanzhou Affiliated to Fujian Medical University, together with the module for patients' informed consent.

### 2.2. Eligibility Criteria

Inclusion criteria are as follows: age ≥ 60, treatment-naive AMI patients meeting the diagnostic criteria of AMI [12], and Killip classification II-III. Exclusion criteria are as follows: severe primary organ diseases of the heart, liver, or kidney, essential hypertension, or coagulopathy; cognition disorders and severe peripheral nerve or central nervous system diseases; old myocardial infarction; those who refused to accept PCI; local or systemic infectious diseases; and incomplete clinical data.

### 2.3. Nursing Methods

#### 2.3.1. In All Patients, Emergency PCI Was Performed by the Same Surgeon, Followed by 3 Months of Nursing

The Con received routine care, mainly including keeping the ward quiet, maintaining appropriate temperature and humidity, giving healthy dietary guidance, asking patients to stop smoking and limit alcohol, controlling diet, and adjusting personal emotions. In addition, the nursing staff paid attention to the changes in the drip rate and related precautions as well as patients' vital signs during intravenous injection. Patients were also monitored to take preventive drugs for AMI and informed of the causes and predisposing factors of AMI.

The Res was intervened by the CNP model, with the primary approaches as follows.

1. Formulation of a reasonable CNP. The clinical medical staff jointly set up a nursing pathway group to comprehensively assess each patient's condition to formulate a scientific and reasonable nursing pathway, which mainly included health publicity and education, diet nursing, and psychological nursing [13]. In order to get the active cooperation of patients and their families, nurses introduced the contents and necessity of the pathway in detail and carried out evaluation according to the specific clinical condition of patients
2. Implementation of CNP. The green first aid channel was refined. Five minutes before the patient's arrival, the medical staff got prepared to receive the patient in the emergency center and immediately sent the patient to the emergency room upon the patient's arrival. Then, the patient's condition was immediately reassessed, and corresponding physical examination, blood tests, etc. were performed. After the contraindication of thrombolysis was excluded and the diagnosis of myocardial infarction (MI) was confirmed, the patient's family members' informed consent was got after informing them about the treatment risks. Thrombolytic care: considering that patients were at high risk during intravenous thrombolytic therapy, professionals were there to accompany and guard patients and to control the infusion speed and time. Besides, the venous access was kept unimpeded, the patient's condition was strictly observed, and any abnormal conditions were handled in time to avoid serious adverse events. On the day of admission, the nursing staff actively communicated with the patient, introduced the relevant precautions, and carefully examined the patient's clinical symptoms. In addition, nurses took the initiative to introduce the hospital environment, medical conditions, and related management procedures to patients and listened to the patient to understand his/her relevant information, so as to implement an effective assessment. From the second day of admission to the day before discharge, the nursing staff took corresponding measures to actively give health guidance to patients, including the cause of the disease, diagnosis and treatment methods, and matters needing attention, so that they can quickly understand the disease. What is more, patients were guided to carry out routine examinations, and their psychological changes were observed, so as to take targeted psychological care to avoid negative emotions such as anxiety and uneasiness. Meanwhile, the nursing staff actively guided patients to eat and train, so as to make them aware of the importance of reasonable diet and physical exercise, thereby enhancing immunity and treatment compliance. Upon discharge from hospital, the nursing staff informed the patient of regular review according to the doctor's advice, so that the patient can grasp the cure of the disease in time. At the same time, health education for discharge was strengthened, which mainly included medication guidance, namely, strictly following the doctor's advice to take drugs, so that patients can master the correct medication methods
3. The CNP team summarized and evaluated the daily implementation and analyzed the possible problems or deficiencies in the nursing process, so as to make corresponding adjustments in time. During the whole nursing process, the CNP leader or head nurse randomly checked the implementation of patients' nursing measures and investigated the nursing satisfaction before patients were discharged from hospital

### 2.4. Endpoints

#### 2.4.1. Primary Endpoints

*(1) Overall Response Rate (ORR)*. Efficacy evaluation criteria are as follows: markedly effective: the clinical symptoms were resolved, with examination results indicating significantly improved cardiac function; effective: the clinical symptoms were resolved to some extent, with examination results indicating some certain cardiac function improvement; and ineffective: no improvement in clinical symptoms nor in cardiac function. ORR = (markedly effective + effective) cases/total cases × 100%.

*(2) Incidence of Complications*. The incidence of complications (arrhythmia, chest pain, cardiogenic shock, constipation, etc.) was calculated.

*(3) Clinical Efficacy Indicators*. The total emergency treatment time, hospitalization, medical expenses, and recurrence rate of MI were recorded to evaluate the clinical efficacy.

*(4) Cardiac Function Indexes (N-Terminal Pro-Brain Natriuretic Peptide (NT-Pro BNP) and Left Ventricular Ejection Fraction (LVEF))*. Fasting venous blood was sampled before and after treatment to determine NT-pro BNP levels by ELISA, strictly following the instructions of human NT-pro BNP ELISA kits (Shanghai Hengfei Biotechnology Co., Ltd., Shanghai, China, SEKH-0112).

#### 2.4.2. Secondary Endpoints

1. Patients' adverse moods such as anxiety and depression before and after nursing intervention were scored using the Self-rating Anxiety/Depression Scale (SAS/SDS) [14], respectively. Both scales have a total score of 100 points, with a score of 50-70, 71-90, and >90 indicating mild, moderate, and severe anxiety/depression, respectively. Higher scores were associated with increased severity of anxiety/depression
2. Patients' QOL were assessed using the Generic Quality of Life Inventory-74 (GQOLI-74) [15] from four dimensions of physical function, social function, psychological function, and material life function, with higher scores suggesting better QOL
3. Patients were scored by the self-made nursing satisfaction questionnaire for their nursing satisfaction after intervention. A total of 20 questions (5 points each) were scored by patients according to the nursing contents, with a total score of <70, 70-89, and ≥90 indicating dissatisfied, satisfied, and very satisfied, respectively. Satisfaction was calculated as the number of cases who were very satisfied and satisfied divided by the total cases

### 2.5. Statistical Processing

Data analysis and image rendering were done by SPSS24.0 (IBM Corp., Armonk, NY, USA) and GraphPad Prism 7, respectively. Counting data, recorded as [*n*(%)], were compared using the chi-square test. Measurement data were given as the mean ± standard deviation (*x* ± SD) and compared by the independent samples *t*-test between groups and paired *t*-test before and post treatment within the group. *P* < 0.05 was the significance level for all tests.

## 3. Results

### 3.1. General Data

The two groups were similar in general clinical baseline data like gender, age, body mass index (BMI), Killip classification, marital status, residence, educational background, and smoking, drinking, hypertension, and diabetes history (*P* > 0.05) (Table 1).

### 3.2. ORR

After nursing intervention, the ORR was 91.84% in the Res and 81.01% in the Con, with statistical significance (*P* < 0.05) (Table 2).

### 3.3. Incidence of Complications

After nursing intervention, the incidence of complications was 5.10% in the Res and 15.19% in the Con, with statistical significance (*P* < 0.05) (Table 3).

### 3.4. Clinical Efficacy Indexes

After nursing intervention, the time of total emergency treatment and hospitalization and the medical expenses and recurrence rate of MI were notably lower in the Res versus the Con (*P* < 0.05) (Table 4).

### 3.5. Cardiac Function Indexes

The levels of LVEF and NT-pro BNP were not statistically different between groups before intervention. After intervention, LVEF of the two groups increased while NT-pro BNP level decreased, and the increase in LVEF and the decrease in NT-pro BNP were more significant in the Res compared with the Con (*P* < 0.001) (Figure 1).

### 3.6. SAS and SDS Scores

SAS and SDS scores were not statistically different between groups before nursing intervention (*P* > 0.05). After nursing intervention, both scores were significantly reduced, with lower scores in the Res compared with the Con (*P* < 0.001) (Figure 2).

### 3.7. GQOLI-74 Scores

In terms of QOL, patients in the Res scored higher in physical function, social function, psychological function, and material life function than those in the Con after nursing intervention (*P* < 0.05) (Figure 3).

### 3.8. Comparison of Nursing Satisfaction

The Res outperformed the Con in nursing satisfaction after nursing intervention (93.88% vs. 79.75%, *P* < 0.05) (Table 5).

## 4. Discussion

AMI in the elderly is a common and frequently occurring disease in clinical cardiovascular medicine [16, 17]. Today, accelerated population aging has driven the constantly rising incidence of AMI and its increasing prevalence at younger ages; moreover, the disease progresses rapidly, which poses a serious impact on patients' physical and mental health and QOL and increases their economic burden [18]. Emergency PCI is the first choice to treat AMI, but due to the decline of patients' body function to varying degrees, it is prone to bring adverse effects on patients' mood and behavior, causing psychological problems such as preoperative anxiety and depression, thus affecting the efficacy of clinical treatment and nursing [19–21]. Routine nursing only focused on saving patients' lives, but ignored the changes of patients' emotional and psychological state, which affected patients' QOL [22, 23]. Herein, we investigated the impact of CNP intervention on the efficacy and QOL of elderly AMI patients.

Zhang et al. [24] reported that the modified early warning score combined with CNP can improve the clinical efficacy of first aid for AMI patients and reduce the incidence of complications. This research found that the ORR was significantly higher and the complication rate was markedly lower in the Res versus the Con, indicating that CNP contributes to significantly enhanced treatment effects and reduced postoperative complications, which agreed with the study of Zhang et al. We also compared the time of total emergency treatment and hospitalization, as well as the hospitalization expenses and recurrence rate of MI between the two groups. The results revealed better parameters in the Res, which indicated that the intervention measures of CNP could significantly reduce the first aid time, LOS, and costs of patients and effectively reduce the recurrence rate of MI. This may be because the implementation of CNP enables patients to have a higher awareness of the disease and the nursing content, which mobilizes patients to better cooperate with the work of medical staff and consequently effectively improve the ability of medical staff to deal with complications and emergencies, ultimately improving the overall efficacy and prognosis of patients. Zhang et al. [25] found that CNP intervention after PCI can significantly reduce hospital admission time, hospitalization expenses, LOS, and postoperative complications and improve patients' satisfaction with treatment, which was similar to our research results. According to Li and Liu [26], the implementation of CNP intervention following PCI can significantly relieve patients' bad mood and improve their QOL. In the present study, we found significantly lower SAS and SDS scores in the Res, indicating that CNP can effectively mitigate patients' anxiety and depression and improve their mental health, which was similar to the study of Li and Liu. The reason behind this may be that the implementation of the CNP allows patients to grasp the relevant content of care in a timely manner, and greatly improves the relationship between doctors and patients, which is conducive to timely understanding and intervention of patients' psychological state, thus mitigating their adverse emotions. Further, we compared the cardiac function indexes of patients and identified significantly higher LVEF levels and statistically lower NT-pro BNP levels in the Res, suggesting that the implementation of CNP can effectively improve patients' cardiac function indexes. It may be that CNP can exercise the postoperative function of patients and pays close attention to the intervention of patients' psychological state. Li et al. [27] revealed that the structured team nursing model was helpful to shorten the treatment time of patients with MI undergoing PCI, improve their cardiac function, exercise endurance, self-care ability, and QOL, and reduce the occurrence of complications, which is similar to our research findings. Finally, comparisons of patients' QOL and nursing satisfaction identified markedly higher QOL scores and nursing satisfaction in the Res compared with the Con, indicating that CNP can validly improve patients' postoperative QOL as well as nursing satisfaction. Similarly, Zhou et al. [28] found that the application of evidence-based nursing in patients with AMI can significantly improve patients' cardiac function, QOL, and nursing satisfaction.

## 5. Conclusion

While significantly enhancing clinical efficacy and reducing complications, CNP intervention for elderly patients with AMI can improve their cardiac function, relieve bad emotions, and improve QOL and nursing satisfaction. However, this study still shows deficiencies. First, analysis of the risk factors affecting postoperative rehabilitation can be supplemented to provide a basis for patients' prognosis assessment. In addition, we can extend the follow-up time to explore the long-term intervention effect of this model on patients. Moreover, the prospect of this nursing model is very considerable, and we can constantly update and improve its nursing concept and measures. We will address the deficiencies in future research to improve our research.

## Figures and Tables

**Figure 1:** Comparison of cardiac function indexes. In comparison with the Con, LVEF (a) of patients was higher while NT-pro BNP (b) was lower in the Res after nursing intervention. ^∗∗∗^*P* < 0.001 vs. before nursing (paired *t*-test); ^∗∗∗^*P* < 0.001 vs. the Con after nursing (*t*-test).

**Figure 2:** Comparison of SAS and SDS scores. After nursing intervention, SAS scores (a) and SDS scores (b) decreased significantly in both groups, with more significant decreases in the Res. ^∗∗∗^*P* < 0.001 vs. before nursing (paired *t*-test); ^∗∗∗^*P* < 0.001 vs. the Con after nursing (*t*-test).

**Figure 3:** Comparison of GQOLI-74 scores between two groups. After nursing intervention, the Res scored higher in physical (a), social (b), mental (c), and material life function (d) than the Con. ^∗∗∗^*P* < 0.001 vs. the Con after nursing (*t*-test).

**Table 1:** Comparison of general information ([*n*(%)], *x* ± SD).

Classification	The Res (*n* = 98)	The Con (*n* = 79)	*t*/*χ*^2^ value	*P* value
Gender			0.007	0.928
Male	54 (55.10)	43 (54.43)		
Female	44 (44.90)	36 (45.57)		
Age (years old)	66.02 ± 3.82	65.54 ± 3.74		
BMI (kg/m^2^)	22.68 ± 2.02	22.82 ± 2.18		
Killip classification			0.177	0.673
Class II	65 (66.33)	50 (63.29)		
Class III	33 (33.67)	29 (36.71)		
Marital status			0.033	0.854
Married	72 (73.47)	59 (74.68)		
Single	26 (26.53)	20 (25.32)		
Residence			0.003	0.949
Urban	60 (61.22)	48 (60.76)		
Rural	38 (38.78)	31 (39.24)		
Educational background			0.314	0.575
≥ High school	43 (43.88)	38 (48.10)		
< High school	55 (56.12)	41 (51.90)		
History of smoking			0.208	0.647
Yes	46 (46.94)	34 (43.04)		
No	52 (53.06)	45 (56.96)		
History of drinking			0.064	0.799
Yes	69 (70.41)	57 (72.15)		
No	29 (29.59)	22 (27.85)		
History of hypertension			0.080	0.776
Yes	50 (51.02)	42 (53.16)		
No	48 (48.98)	37 (46.84)		
History of diabetes			0.028	0.865
Yes	36 (36.73)	30 (37.97)		
No	62 (63.27)	49 (62.03)		

**Table 2:** Comparison of overall response rate after nursing intervention [*n*(%)].

Groups	Effective	Markedly effective	Ineffective	Overall response rate
The Res (*n* = 98)	75 (76.53)	15 (15.31)	8 (8.16)	90 (91.84)
The Con (*n* = 79)	36 (45.57)	28 (35.44)	15 (18.99)	64 (81.01)
*χ* ^2^	—	—	—	4.533
*P*	—	—	—	0.030

**Table 3:** Comparison of complication rate after nursing intervention [*n*(%)].

Groups	Arrhythmia	Chest pain	Cardiogenic shock	Constipation	Total incidence
The Res (*n* = 98)	1 (1.02)	2 (2.04)	0 (0.00)	2 (2.04)	5 (5.10)
The Con (*n* = 79)	3 (3.80)	3 (3.80)	2 (2.53)	4 (5.06)	12 (15.19)
*χ* ^2^	—	—	—	—	5.127
*P*	—	—	—	—	0.023

**Table 4:** Comparison of clinical efficacy indexes after nursing intervention (*x* ± SD).

Groups	Total emergency treatment time (min)	Hospital stay (d)	Medical expenses (CNY)	Recurrence rate of myocardial infarction (%)
The Res (*n* = 98)	25.70 ± 3.40	14.93 ± 1.09	7735.74 ± 216.33	5.10
The Con (*n* = 79)	36.36 ± 4.53	23.09 ± 1.31	9845.86 ± 375.20	21.52
*t*/*χ*^2^	17.880	45.230	46.860	10.830
*P*	<0.001	<0.001	<0.001	0.001

**Table 5:** Comparison of nursing satisfaction [*n*(%)].

Classification	The Res (*n* = 98)	The Con (*n* = 79)	*χ* ^2^ value	*P* value
Very satisfied	70 (71.43)	30 (37.98)	—	—
Satisfied	22 (22.45)	33 (41.77)	—	—
Dissatisfied	6 (6.12)	16 (20.25)	—	—
Nursing satisfaction	92 (93.88)	63 (79.75)	8.024	0.004

## Data Availability

The simulation experiment data used to support the findings of this study are available from the corresponding author upon request.
